The article "Identification of ATG7 as a Regulator of Proferroptosis and Oxidative Stress in Osteosarcoma" was retracted in 2023. Reasons: unreliable results or conclusions; concerns about the data; concerns about the peer review; concerns about the citations.

# Identification of ATG7 as a Regulator of Proferroptosis and Oxidative Stress in Osteosarcoma

**DOI:** 10.1155/2022/8441676

**Published:** 2022-10-08

**Authors:** Runyi Jiang, Shaohui He, Haiyi Gong, Yao Wang, Wei Wei, Jun Chen, Jinbo Hu, Chen Ye, Shuchen LiuHuang, Saiying Jin, Haifeng Wei, Wei Xu, Jianru Xiao

**Affiliations:** ^1^Spinal Tumor Center, Department of Orthopaedic Oncology, Changzheng Hospital, Second Military Medical University, Shanghai 200003, China; ^2^Department of Orthopaedic Surgery, No. 905 Hospital of PLA Navy, Second Military Medical University, Shanghai 200050, China; ^3^Department of Pathology, Changzheng Hospital, Second Military Medical University, Shanghai 200003, China; ^4^School of Medical Instrument and Food Engineering, University of Shanghai for Science and Technology, Shanghai 200093, China; ^5^School of Design and Innovation, China Academy of Art, Hangzhou, China

## Abstract

**Background:**

Ferroptosis has gained significant attention from oncologists as a vital outcome of oxidative stress. The aim of this study was to develop a prognostic signature that was based on the ferroptosis-related genes (FRGs) for osteosarcoma patients and explore their specific role in osteosarcoma.

**Methods:**

The training cohort dataset was extracted from the Therapeutically Applicable Research to Generate Effective Treatments (TARGET) database. Different techniques like the univariate Cox regression, least absolute shrinkage and selection operator (LASSO) regression, multivariate Cox regression analyses, and the Kaplan-Meier (KM) survival analyses were utilized to develop a prognostic signature. Then, the intrinsic relationship between the developed gene signature and the infiltration levels of the immune cells was further investigated. An external validation dataset from the Gene Expression Omnibus (GEO) database was employed to assess the predictive ability of the developed gene signature. Subsequently, the specific function of potential FRG in affecting the oxidative stress reaction and ferroptosis of osteosarcoma cells was identified.

**Results:**

A prognostic signature based on 5 FRGs (CBS, MUC1, ATG7, SOCS1, and PEBP1) was developed, and the patients were classified into the low- and high-risk groups (categories). High-risk patients displayed poor overall survival outcomes. The risk level was seen to be an independent risk factor for determining the prognosis of osteosarcoma patients (*p* < 0.001, hazard ratio: 7.457, 95% CI: 3.302-16.837). Additionally, the risk level was associated with immune function, which might affect the survival status of osteosarcoma patients. Moreover, the findings of the study indicated that the expression of ATG7 was related to the regulation of oxidative stress in osteosarcoma. Silencing the ATG7 gene promoted the proliferation and migration in osteosarcoma cells, suppressing the oxidative stress and ferroptosis process.

The article "Identification of ATG7 as a Regulator of Proferroptosis and Oxidative Stress in Osteosarcoma" was retracted in 2023. Reasons: unreliable results or conclusions; concerns about the data; concerns about the peer review; concerns about the citations.

**Conclusions:**

A novel FRG signature was developed in this study to predict the prognosis of osteosarcoma patients. The results indicated that ATG7 might regulate the process of oxidative stress and ferroptosis in osteosarcoma cells and could be used as a potential target to develop therapeutic strategies for treating osteosarcoma.

## 1. Introduction

Osteosarcoma (OS) is reported to be a very prevalent type of malignant bone tumor affecting children and teenagers, and it has an annual incidence rate of 4.4 per million people [1]. With the advent of chemotherapy, the prognosis of patients with localized OS has substantially improved, with the long-term overall survival rate increasing from <20% to 65-70% [2, 3]. However, survival outcomes for patients with metastases and those who poorly responded to initial treatment are still low, with an estimated 5-year survival rate of ~25% for patients aged between 2 and 68 years [4]. The role of common regulated cell death (RCD) processes, such as autophagy and apoptosis, in treating OS patients is still controversial [5, 6]. Therefore, it is crucial to seek other novel and efficient approaches to OS treatments.

One of the key distinguishing features of tumor cells is their high energy metabolism [7]. Reactive oxygen species (ROS) are commonly generated accompanied by increased metabolism, which causes oxidative stress in tumor cells [8]. Generally, the balance of ROS is crucial for normal cell growth and survival [9]. High ROS produces DNA damage which further leads to more mutations and initiation of cancers [10, 11]. In addition, high ROS also causes lipid, protein, and DNA damage to normal cells, often leading to apoptosis [12, 13]. However, the apoptotic machinery is damaged in cancer cells as well, which results in more tumor cell proliferation in turn [9]. The studies on ROS are vast and controversial. Since ROS plays a vital role in the onset and progression of tumors, regulating the antioxidative stress in tumor cells might open a new direction for treating tumors.

Ferroptosis, which is a Fe-dependent form of RCD that is activated by excessive lipid peroxidation due to the lethal accumulation of ROS, attracted the attention of many oncologists [14]. In comparison to the noncancerous cells, the tumor cells display an increased Fe demand to enable growth [15], and ROS is an important product of metabolism in cancer cells [7]. Studies have shown that ferroptosis could be induced in OS cells by experimental reagents (such as erastin and RSL3) through extrinsic or intrinsic pathways [16–18]. In addition, sorafenib, a drug reported to induce ferroptosis, suppresses tumor growth, angiogenesis, and metastatic potential in OS cells [19]. These findings provided the theoretical foundation for OS treatments by inducing ferroptosis by altering the oxidative stress balance in OS cells. Thus, therapy targeting ferroptosis-related genes (FRGs) might be a novel way to treat OS, especially metastatic and insensitive to initial treatment patients. Although ferroptosis is observed to play a vital role in different malignant or benign tumors [20, 21], their specific function and prognostic values in OS remain largely unknown.

The article "Identification of ATG7 as a Regulator of Proferroptosis and Oxidative Stress in Osteosarcoma" was retracted in 2023. Reasons: unreliable results or conclusions; concerns about the data; concerns about the peer review; concerns about the citations.

In this report, the RNA sequencing results and the corresponding clinical data of the OS patients were downloaded from the Therapeutically Applicable Research to Generate Effective Treatments (TARGET) database. Then, the expression of the FRGs was analyzed in OS patients, and a novel prognostic multigene signature was generated that was based on the FRGs derived from the TARGET cohort. Then, its prognostic significance was verified using a Gene Expression Omnibus (GEO) cohort. Moreover, the potential role of candidate FRG in oxidative stress and tumor development in OS cells was validated by experiments. The results of this study have yielded an FRG that could potentially be used as a therapeutic target for developing effective strategies to treat OS.

## 2. Materials and Methods

### 2.1. Data Collection

RNA sequencing data and the related clinical information of 101 OS patients were obtained from the TARGET cohort (https://ocg.cancer.gov/programs/target, Figure S1). The following inclusion criteria were used for further screening: (1) OS patients with confirmed survival status and active follow-up, (2) survival time > 0 months, and (3) complete information of metastatic status in the clinical records. The exclusion criteria were as follows: (1) patients with missed follow-ups, (2) unknown or 0 survival months, and (3) duplicate samples. Among those, 93 OS patients were finally included in the training cohort for further study, and the RNA sequencing data of these patients were normalized to transcripts per million (TPM) values before analyses. In addition, the GSE21257 sequence (Platform GPL10295) was retrieved from the Gene Expression Omnibus (GEO) cohort (https://www.ncbi.nlm.nih.gov/geo/query/acc.cgi?acc= GSE21257) as the validation dataset. This dataset comprised 53 OS patients, including 34 (64.1%) samples with metastasis and 19 (35.9%) samples without metastasis. 200 FRGs were analyzed in this study (Table S1).

The article "Identification of ATG7 as a Regulator of Proferroptosis and Oxidative Stress in Osteosarcoma" was retracted in 2023. Reasons: unreliable results or conclusions; concerns about the data; concerns about the peer review; concerns about the citations.

### 2.2. Identification of Osteosarcoma Subclusters

The nonnegative matrix factorization (NMF) was performed after a filtering procedure using the R package “NMF” to cluster the obtained FRGs. Candidate genes with mean expression < 0.05 were discarded. The selected FRGs were then subjected to a univariate Cox regression analysis to assess the correlation between the selected candidate genes and the survival rate using the “survival” R package. Genes with *p* < 0.05 were chosen for sample clustering.

### 2.3. Designing and Validating the Prognostic Model Based on FRGs

The Kaplan-Meier (KM) curves were used to decipher the significant prognostic FRGs using the results of the univariate Cox regression analysis (*p* < 0.05), and genes with *p* ≤ 0.01 were subjected to the least absolute shrinkage and selection operator (LASSO) regression analysis. R packages like “survminer” and “glmnet” were used for these analytical techniques, respectively. LASSO regression is excellent for narrowing down the candidate genes and minimizing the risk of overfitting [22]. Ultimately, the results of LASSO regression were included in the multivariate Cox regression analysis, and the *β* value (the regression coefficient of each gene integrated within this model) was evaluated for each FRG. This was used for developing the formula for estimating the risk score for patients.

(1) $$\begin{array}{c} \text{Risk score}=\overset{n}{\underset{i}{\sum }}\left({\text{Coefficient}}_{\text{mRNA}i}*{\text{Expression}}_{\text{mRNA}i}\right). \end{array}$$

Individuals were classified into the low- and high-risk subgroups (categories) based on their median risk scores, and the likelihood of survival was compared between both groups. The “survivalROC” R package was used to create the receiver operating characteristic (ROC) curves, which were then used to calculate the performance score of the developed FRG signature models based on the area under the ROC curves (AUC-ROC). Finally, the predictive power of the developed model was evaluated using Harrell's concordance index (*C*-index). Following a reordering of the subjects according to their risk scores, the risk curves, the survival status-based scatterplot, and heatmap of the expression of FRGs were plotted. For additional validation, the GSE21257 cohort was obtained from the GEO database. Briefly, the “scale” function was used for the purpose of normalizing the expression level of every FRG expression in the external cohort, and the same procedure was used to determine risk scores for the validation cohort. Using the ideal cutoff value, patients included in the GSE21257 dataset were also divided into the low- or high-risk subgroups to confirm the accuracy of the developed model.

The article "Identification of ATG7 as a Regulator of Proferroptosis and Oxidative Stress in Osteosarcoma" was retracted in 2023. Reasons: unreliable results or conclusions; concerns about the data; concerns about the peer review; concerns about the citations.

### 2.4. Independent Prognostic Analysis by Incorporating the “Risk Score”

The “risk score,” a binary variable (low-/high-risk group) as a new potential factor, were combined with other clinical features to build a new dataset for further prognostic analysis. The univariate and multivariate Cox regression analyses were used to determine the significant prognostic clinical factors. Factors having a *p* value < 0.05 of both the Cox regression analyses were included to develop a nomogram, with the help of the R-package “rms” to anticipate the survival likelihood of the OS patients. Factors like AUC, *C*-index, and calibration curves were used to assess the accuracy of the generated nomogram, and ROC curves of each clinical factor and decision curve analysis (DCA) were employed to determine if the risk level could be utilized as an independent prognostic factor.

### 2.5. Gene Ontology (GO) Analyses and Immune Signature of the Subgroups

The differentially expressed genes (DEGs) existing in the high- and low-risk subgroups in the training dataset were extracted using the “limma” package. Genes with adjusted *p* value < 0.05 and absolutelog_2_FC ≥ 1 were considered DEGs and subjected to GO enrichment analyses by applying the “ClusterProfiler” package.

Furthermore, the immune cell types in two subgroups were evaluated by TIMER2.0 (http://timer.cistrome.org), and the activity of the 13 immune-linked functions was determined with single-sample gene set enrichment analysis (ssGSEA) using the “GSVA” R package. Furthermore, immune checkpoint gene analysis was also carried out to ascertain ferroptosis-linked potential immune checkpoint genes. Functional analyses were also carried out using the validation dataset.

### 2.6. Exploration of the Relationship between ATG7 and Oxidative Stress in OS

Patients were categorized into 2 subgroups based on the optimal cut-off value of the ATG7 expression. DEGs between both groups could be identified using the above criteria. GO enrichment analyses were then performed to examine the differences between both groups. Additionally, ssGSEA was utilized to assess the differences (variations) in the oxidative stress pathways that were differentially expressed in the ATG7 groups.

### 2.7. Cell Culture

OS cell lines (MG63, HOS) and the human bone marrow mesenchymal stem cells (hBMSC) were procured from the National Collection of Authenticated Cell Cultures (Shanghai, China). The MG63 and HOS cell lines were cultured using DMEM, while the hBMSC lines were cultured in *α*-MEM. All the media were supplemented with fetal bovine serum (10% *v*/*v*) (FBS, Gibco) and the penicillin/streptomycin solution (P/S, 100 U/ml, Gibco). All cell lines were cultured in the humidified carbon dioxide incubator (5% CO_2;_ 37°C temperature).

The article "Identification of ATG7 as a Regulator of Proferroptosis and Oxidative Stress in Osteosarcoma" was retracted in 2023. Reasons: unreliable results or conclusions; concerns about the data; concerns about the peer review; concerns about the citations.

### 2.8. ATG7 RNA Interference

The OS cell line, MG63, was cultured in 6-well culture plates until they achieved a 60% confluency before the cells were transfected with ATG7-RNAi (3 *μ*l, 40 pmol) in a serum-free medium, in the presence of lipofectamine 3000 (2 *μ*l, Thermo, USA), based on the manufacturer's instructions. After incubating the transfection mixture for 6 h, MG63 cells were maintained in a fresh medium. After 48 h, the Western blotting (WB) technique was used to test the effects of ATG7 gene silencing. siRNAs for ATG7 (siATG7-1: GCCTGCTGAGGAGCTCTCCAT; siATG7-2: CCTAAAGAAGTACCACTTCTA) and the negative siRNA control (siNC) were synthesized by the Genepharm Technologies (Shanghai, China).

### 2.9. Cell Viability and Migration

The siATG7-transfected MG63 cells were seeded into the 96-well culture plates. Cell viability was assessed using the Cell Counting Kit-8 (CCK8) reagent (Vazyme, A311-02-AA) based on the kit instructions. All the cells were incubated with the CCK8 reagent for 60 min at a temperature of 37°C, and the absorbance values (450 nm) were noted at differing time points (days 1, 2, 3, and 4). Moreover, the CellTiter-Glo luminescent Cell Viability Assay (G7572, Promega, USA) was used to test the viability of the MG63 cells that were treated using the RSL3 (10 *μ*M), a ferroptosis inducer (Selleck, S8155), after silencing the ATG7 gene. These cells recorded the luminescence at various time points (0, 12, 24, and 48 h) [23].

Cells, in the logarithmic growth phase, were cultured into the 6-well culture plates for a minimum of 7 days and stained using 0.1% (*v*/*v*) crystal violet for conducting the colony formation assay. Using the Transwell chambers (pore size: 8 mm, Corning), the cells were resuspended in the serum-free medium (200 *μ*l) and placed in the upper chamber for performing the migration tests. The lower chambers were then filled with the DMEM (500 *μ*l), supplemented with FBS (10% *v*/*v*), and incubated for 24 h. The cells were then stained using 0.1% (*v*/*v*) crystal violet after being fixed with 4% (*v*/*v*) paraformaldehyde. The Image-Pro Plus 6.0 software was used for counting the migrating cells, and the bright-field images were captured using an Olympus inverted microscope (Media Cybernetics, USA).

### 2.10. Determining the Malondialdehyde (MDA), Superoxide Dismutase (SOD), and Lipid ROS Concentrations

MDA concentration was measured following kit instructions (Beyotime, S0131S). In addition, the cells were stained using C11-BODIPY (D3861, Thermo Fisher Scientific, USA), followed by flow cytometry to measure the lipid ROS production [24]. SOD activity was measured using the WB technique. It is noteworthy that the ATG7-silenced MG63 cells should undergo RSL3-induced ferroptosis for about 12 h before all measurements.

The article "Identification of ATG7 as a Regulator of Proferroptosis and Oxidative Stress in Osteosarcoma" was retracted in 2023. Reasons: unreliable results or conclusions; concerns about the data; concerns about the peer review; concerns about the citations.

### 2.11. Iron Accumulation

The level of iron in the MG63 cells was measured in two ways. One tested the free ferrous iron (Fe^2+^) using a commercial Fe assay kit (ab83366, Abcam) based on the kit instructions, and in another technique, the expression of FTH1 was tested following the WB technique. RSL3-induced ferroptosis (12 h) was also implemented in MG63 cells transfected with siATG7 before measuring.

### 2.12. Quantitative Real-Time Polymerase Chain Reaction (qPCR) and Western Blotting Techniques

Total RNA was extracted with the help of the TRIzol reagent (Thermo Fisher Scientific, Waltham, MA, USA). Reverse transcription and qPCR techniques were performed utilizing the PrimeScript™ RT Master Mix and SYBR Premix ExTaq (Takara, Kyoto, Japan), based on the kit instructions. The data were assessed using the 2^-*ΔΔ*Ct^ technique.

Total proteins were extracted using the RIPA buffer, then loaded uniformly onto the SDS-PAGE (sodium dodecyl sulfate, 10%) gel, and transferred to the nitrocellulose membranes. The membranes were then blocked with bovine serum albumin (BSA, 5%) and incubated with the primary antibodies such as anti-FTH1 (ABclonal, A19544), anti-SOD (Cell Signaling Technology, 71G8), anti-ATG7 (Abcam, ab52472), and anti-GAPDH (Sigma-Aldrich, USA). Thereafter, the membranes were washed and incubated with horseradish peroxidase- (HRP-) conjugated secondary antibodies. Finally, the membranes were washed and imaged using the ChemiDoc XRS+ System (Bio-Rad Laboratories, USA).

### 2.13. Statistical Analysis

All the data were statistically analyzed using R software (ver. 4.0.1) and GraphPad Prism 8.0. All the quantitative data were expressed as mean standard deviation (SD), whereas the categorical variables were presented using counts and percentage values. Wilcox test was employed to detect the DEGs and evaluate the GO enrichment and immune-linked functions, whereas the log-rank test was employed to analyze the overall survival rate of OS patients. The *t*-test was used to examine the findings of the experiments. Each experiment was carried out at least 3 times, with representative findings. Differences with a two-tailed *p* < 0.05 were considered statistically significant (^∗^*p* < 0.05, ^∗∗^*p* < 0.01, and ^∗∗∗^*p* < 0.001).

## 3. Results

### 3.1. Identification of OS Subclusters Based on FRGs

A total of 200 candidate FRGs were initially obtained from the RNA-seq dataset training cohort. The univariate Cox regression results revealed that 26 FRGs (including 7 risk and 19 protective genes) fulfilled the inclusion criteria and were depicted in the forest plot (Figure 1(a)). NMF was performed to determine potential characteristics in the gene expression profiles by decomposing the initial matrix into 2 nonnegative matrices [25]. The 26 FRGs were then subjected to the NMF analysis. The 93 OS were categorized into two clusters depending on the optimum *k* value, based on their correlation coefficient values (Figures 1(b), S2A). The consensus matrix heatmap exhibited a sharp and clear boundary, illustrating that the samples had robust and stable clusters with *k* = 2. Consensus matrix heatmaps of other *k* values (*k* = 3-6) are shown in Figure S2B. The differential expression of the 26 FRGs between the two subclusters is shown in the heatmap pattern (Figure 1(c)). The KM curves indicated a significant difference in overall survival for patients between the identified clusters (*p* < 0.0001, Figure 1(d)).

The article "Identification of ATG7 as a Regulator of Proferroptosis and Oxidative Stress in Osteosarcoma" was retracted in 2023. Reasons: unreliable results or conclusions; concerns about the data; concerns about the peer review; concerns about the citations.

### 3.2. Development of Prognostic Gene Signature Using the Training Cohort

Out of the 26 FRGs identified in the univariate analysis, the KM analysis demonstrated that 19 FRGs satisfied the set criteria of *p* ≤ 0.01 and hence were selected for additional analysis. Using the LASSO regression analysis, multivariate Cox regression was applied to 12 FRGs based on their optimal *λ* values (Figures 2(a) and 2(b)). Finally, 5 FRGs were identified to construct a prognostic FRG signature (Figure 2(c)), containing 2 risk FRGs (CBS, MUC1) and 3 protective FRGs (ATG7, SOCS1, and PEBP1). The risk scores were estimated following formula as follows: Risk score = (−0.9427^∗^ATG7 exp.) + (0.4763^∗^CBS exp.) + (0.2692^∗^MUC1 exp.) + (−0.4567^∗^SOCS1 exp.) + (−0.7295^∗^PEBP1 exp.). The *C*-index (0.82) and AUC values for 1-, 2-, and 3-year survival rates of OS patients were 0.758, 0.928, and 0.938, respectively (Figure 2(d)), which indicated the favorable predictive value of this prognostic model. The association of the overall survival rate with the 5 identified FRGs has been shown in Figures 2(e)–2(i). KM curves of the FRGs excluded in the prognostic signature are shown in Figure S3.

Depending on the median risk scores, 93 OS patients were categorized into the low- and high-risk subgroups. The findings revealed a significant difference in the disease prognosis between the 2 categories (*p* < 0.001, Figure 3(a)). Risk curves and scatterplots were generated to demonstrate the risk scores and survival status of every patient (Figures 3(b) and 3(c)), illustrating that the high-risk group patients showed a worse prognosis compared to the low-risk patients. The heatmaps also showed a differential expression of 5 FRGs in the two groups (Figure 3(d)).

The article "Identification of ATG7 as a Regulator of Proferroptosis and Oxidative Stress in Osteosarcoma" was retracted in 2023. Reasons: unreliable results or conclusions; concerns about the data; concerns about the peer review; concerns about the citations.

### 3.3. Independent Prognostic Value of the FRG Signature

Univariate and multivariate Cox regression analyses were used for assessing if the risk level, as the binary variable derived from the risk score, could be used as an independent prognostic factor (Figures 4(a) and 4(b)). The results indicated that metastasis status (*p* < 0.001, HR: 3.656, 95% CI: 1.875–7.131) and risk levels were independent prognostic factors that influenced the overall survival rate of OS patients (*p* < 0.001, HR: 7.457, 95% CI: 3.302–16.837). Additionally, ROC curves and DCA of each clinical factor manifested that risk level was a more robust factor in predicting overall survival rates than any other clinical factor (Figure S4A-B). Depending on the results generated by the multivariate Cox regression analysis, a nomogram was developed to visually evaluate the prognosis of OS patients (Figure 4(c)). Moreover, the *C*-index (0.799), AUC at 1-, 2-, and 3-year survival predictions (Figure 4(d)), and the calibration plots (Figures 4(e)–4(g)) depicted the effectiveness of this nomogram in anticipating the survival status of OS patients.

### 3.4. Functional Analyses of the FRG Risk Model in the Training Cohort

A total of 58 DEGs (adjusted *p* value < 0.05; absolutelog_2_FC ≥ 1) were detected in the high- and low-risk groups, out of which 44 DEGs were downregulated, whereas 14 were upregulated. The results of the GO enrichment analysis demonstrated that the immune response and antigen processing and presentation were the primary biological processes (BPs). At the same time, the MHC protein-related complex was the most abundant cellular component (CCs), while the molecule functions (MFs) were primarily related to the MHC protein complex binding or activity (Figure 5(a)). Moreover, the relationship between immune-related functions and risk scores was investigated. The high- and low-risk groups showed a statistically significant difference in the composition of the immune cells. The low-risk group contained a higher number of immune cells like macrophages, CD4^+^ T cells, CD8^+^ T cells, and natural killer (NK) cells (Figure 5(b)). Similarly, the results showed that the activities of the checkpoint molecules and the immune-related functions were significantly lower in the high-risk OS patients compared to the low-risk OS patients (^∗^*p* < 0.05, ^∗∗^*p* < 0.01, and ^∗∗∗^*p* < 0.001, Figures 5(c) and 5(d)).

### 3.5. External Validation of the FRG Signature

The GSE21257 dataset containing gene and clinical information of 53 OS patients was utilized as an external validation cohort. OS patients were categorized into 2 different risk groups based on their optimized cutoff values. The two risk groups in the validation dataset showed a significant difference in their disease prognosis (*p* < 0.01, Figure 6(a)). Consistently, the risk curve and scatterplots suggested better outcomes for the low-risk group OS patients compared to OS patients in the high-risk groups in the validation dataset (Figures 6(b) and 6(c)). Additionally, in agreement with the training cohort, the risk (CBS, MUC1) and protective genes (ATG7, SOCS1, and PEBP1) from the GSE21257 dataset were primarily expressed in the high- and low-risk categories, respectively (Figure 6(d)). The AUC values of the ROC curves were 0.755, 0.725, and 0.679 for the 1-, 2-, and 3-year overall survival prediction, respectively (Figure 6(e)), which revealed satisfactory feasibility and stability of the constructed FRG signature model. Moreover, a similar distribution pattern was found during the GO enrichment analysis (Figure 7(a)) and immune-related characteristics for the validation cohort (Figures 7(b)–7(d)).

The article "Identification of ATG7 as a Regulator of Proferroptosis and Oxidative Stress in Osteosarcoma" was retracted in 2023. Reasons: unreliable results or conclusions; concerns about the data; concerns about the peer review; concerns about the citations.

### 3.6. Influence of the Differentially Expressed ATG7 on Oxidative Stress in OS

A total of 48 DEGs (18 downregulated and 30 upregulated genes) were found in the low and high expressed ATG7 groups (Figure 8(a)). The DEGs were partly enriched in oxidative stress-related BPs like regulation of hydrogen peroxide-mediated programmed cell death and multiple oxidative stress-related MFs such as oxygen oxidoreductase (deaminating) activity for several compounds. Meanwhile, the expression of ATG7 may affect the activity of the ferritin receptor (Figure 8(b)). In addition, the results showed that the oxidative stress-related pathways like the regulation of oxidative stress response, regulation of the oxidative stress-induced cell death, and the regulation of transcription from the RNA polymerase II promoter in response to the oxidative stress differ significantly between both groups (^∗^*p* < 0.05, ^∗∗^*p* < 0.01; Figure 8(c)).

### 3.7. The Different Expressions of Five FRGs in OS Cells and hBMSC

Consistent with the above findings, qPCR showed that the 2 risk FRGs (CBS and MUC1) were highly expressed in both OS cell lines (MG63, HOS), and the expression of the 3 protective FRGs (SOCS1, PEBP1, and ATG7) was higher in hBMSC (Figure 9(a)). As autophagy played a crucial role in drug resistance in OS and ATG7 was an essential gene in the autophagy family, the ATG7 gene was selected for further experiments. The results of qPCR and WB further showed that ATG7 expression was downregulated in the MG63 cells rather than hBMSC (Figure 9(b)). This evidence was consistent with all the findings noted in the study.

The article "Identification of ATG7 as a Regulator of Proferroptosis and Oxidative Stress in Osteosarcoma" was retracted in 2023. Reasons: unreliable results or conclusions; concerns about the data; concerns about the peer review; concerns about the citations.

### 3.8. ATG7 Suppressed OS Progression via Mediating Oxidative Stress and Ferroptosis

The CCK8 and colony formation assays demonstrated that silencing the ATG7 gene significantly promoted OS cell proliferation capability (^∗∗^*p* < 0.01, ^∗∗∗^*p* < 0.001; Figures 9(c) and 9(d)). At the same time, enhanced migration ability was found in ATG7-knockdown OS cells (^∗∗∗^*p* < 0.001, Figure 9(e)). These findings indicated that the ATG7 gene might inhibit the proliferation and migration capabilities of the malignant OS cells.

Subsequently, it was noted that the ATG7 gene silencing suppressed the increase in MDA activity, especially when the OS cells encountered oxidative stress (^∗∗∗^*p* < 0.001, Figure 10(a)). Similarly, lipid ROS was also reduced when ATG7 was silenced in OS cells (^∗∗∗^*p* < 0.001, Figure 10(b)). In consistency with the above findings, a decrease in the proportion of cell death (^∗∗∗^*p* < 0.001, Figure 10(c)) with a reduction in the Fe^2+^ levels (^∗∗∗^*p* < 0.001, Figure 10(d)) was found in the siATG7 groups. On the other hand, SOD and FTH1 expression levels were significantly elevated in the ATG7-deficient OS cells (Figure 10(e)). These results indicated that silencing ATG7 might suppress oxidative stress and ferroptosis in OS cells.

## 4. Discussion

Increased oxidative stress is closely related to RCD [26]. As a novel RCD process, ferroptosis is seen to play a crucial role in cancer biology and this process was characterized by its unique gene expression, morphology, and molecular pathways [27, 28]. Ferroptosis could be initiated via regulating different intrinsic or extrinsic pathways. The intrinsic pathway was driven by blocking the intracellular antioxidant enzymes (like glutathione peroxidase, GPX4) [14]. However, the extrinsic pathway involved the inhibition of the cell membrane transporters like the cystine/glutamate transporter (also called the system Xc^−^) or by the activation of the iron transporters like lactotransferrin and serotransferrin [29]. Furthermore, a few earlier studies also reported that many clinical drugs could initiate ferroptosis by inhibiting system Xc^−^ or GPX4 [30–32], providing a new way of treating cancer for oncologists. The canonical chemotherapy for OS combines high-dose methotrexate, doxorubicin, and cisplatin (MAP) [2, 33]. However, this strategy poses little effect on drug-resistant, recurrent, or metastatic OS patients [4]. Studies on ferroptosis in bone tumors, especially in OS, are still lacking. Therefore, this study is aimed at exploring the potential effects of the ferroptosis process on OS patients.

In this study, a novel multigene prognostic signature was constructed for OS patients. Gene signature models have been used in the past to predict the prognosis of patients with different types of cancers [34–36]. This study systematically explored the expression of 200 FRGs in OS tumor tissue samples and their associations with patients' overall survival. Similarly, the results of this study indicated that this five-FRG-based signature could be used for classifying OS patients into 2 clusters with different prognoses and molecular characteristics. Interestingly, patients with high expression of protective FRGs seemed to have better prognoses. Therefore, it was hypothesized in this study that ferroptosis might affect OS patients' prognosis, and constructing a prognostic model based on the FRGs for OS patients could be helpful.

The article "Identification of ATG7 as a Regulator of Proferroptosis and Oxidative Stress in Osteosarcoma" was retracted in 2023. Reasons: unreliable results or conclusions; concerns about the data; concerns about the peer review; concerns about the citations.

Although the application of ferroptosis in tumors has been extensively studied in the past, the probable relationship between ferroptosis and tumor immunity needs further investigation. Previous studies have reported that the interferon-gamma (IFN*γ*) molecules secreted from the CD8^**+**^ T cells promoted the ferroptosis and lipid peroxidation processes in the malignant cells [37]. Furthermore, ferroptosis could also modulate the immune function of tumor cells [15]. Moreover, the ferroptosis tumor cells could release distinct ‘find me' signals to recruit some immune cells like the antigen-presenting cells (APCs) to the site of the malignant cells [38]. A few important steps that take place during the interaction between the immune and ferroptosis malignant cells are observed to be phagocytosis and migration, maturation, antigen-processing, and the cross-presentation by DCs [39, 40]. Interestingly, the results of GO enrichment analyses between the 2 risk groups revealed a few unexpected immune-linked biological processes and pathways such as immune cell activation, antigen processing and presenting, and the IFN*γ*-mediated signaling pathways, which were seen to be especially enriched in the low-risk category. Furthermore, the analysis of the immune system suggested that immune-linked activities in the low-risk category were significantly higher than those in the high-risk category, which contributed to a better prognosis in the low-risk group. Taken together, these findings revealed that ferroptosis could be associated with the immune function of the OS patients, benefitting the prognoses of OS patients and indicating that therapeutic strategies that targeted the FRGs could offer a new treatment scheme for OS patients.

Furthermore, the prognostic model that was constructed in this study included 5 FRGs (ATG7, SOSC1, PEBP1, CBS, and MUC1). ATG7 was reported to suppress tumor cell growth in glioma by promoting ferroptosis [41]. The suppressor of cytokine signaling (SOCS) family members are regarded as cytokine signaling inhibitors that regulate cell growth and differentiation. SOCS1 was known as an inhibitor of tumor cell growth [42]. Studies have shown that P53 promoted ferroptosis in tumor cells by blocking the transcription of SLC7A11 and SOCS1 sensitized cells to ferroptosis by controlling P53 target gene expression [43]. Meanwhile, SOCS1 was also a protective FRG and helped in predicting the prognosis of head and neck squamous cell carcinoma patients [44, 45]. In addition, Phosphatidylethanolamine Binding Protein 1 (PEBP1) induced ferroptosis in epithelial cells by generating hydroperoxy-phosphatidylethanolamine [46] and was involved in the cell death process in hepatocellular carcinoma by regulating ferroptosis [47]. PEBP1 was also a robust prognostic marker associated with good outcomes in lung adenocarcinoma [48, 49]. The system Xc^−^/glutathione- (GSH-) GPX4 axis has been considered a primary system in protecting cells from lipid peroxidation-mediated ferroptosis owing to its involvement in eliminating ROS [10]. CBS is the biosynthetic enzyme for cysteine, which is the major component of GSH. CBS overexpression induces ferroptosis resistance in ovarian cancer cells [50]. Additionally, ferroptosis was triggered in hepatocellular carcinoma by suppressing the expression of CBS [51]. Similarly, MUC1 mediates triple-negative breast cancer cells' self-renewal capacity and tumorigenicity by stabilizing system Xc^−^ and inhibits erastin-induced ferroptosis [52]. Moreover, MUC1 was a ferroptosis-related disease marker in nontumor diseases like idiopathic pulmonary fibrosis and ulcerative colitis [53, 54]. In summary, 3 genes in the prognostic signature (ATG7, SOCS1, and PEBP1) were reported to facilitate ferroptosis in tumor cells, while the remaining two genes (CBS, MUC1) are the opposite. Furthermore, the prognoses in the high expressing proferroptotic genes group were better than those in the low-expression group, which were also dramatically opposed to antiferroptotic genes. Therefore, these results provided a significant theoretical basis for the novel FRGs-based prognostic model.

The article "Identification of ATG7 as a Regulator of Proferroptosis and Oxidative Stress in Osteosarcoma" was retracted in 2023. Reasons: unreliable results or conclusions; concerns about the data; concerns about the peer review; concerns about the citations.

Although ferroptosis was distinct from other RCD processes, the potential relationships among them could not be ignored. Autophagy contributes to ferroptosis in cancer cells by ferritin degradation, providing novel insights into the interplay between autophagy and ferroptosis [55]. Notably, autophagy played an essential role in OS chemoresistance, resulting in treatment failure and poor prognosis for OS patients [55–58]. The role of ferroptosis (antitumor) and autophagy (protumor) in OS seem contradictory. Meanwhile, ATG7, as an autophagy-related gene, is critical for the formation of autophagosomes [55]. Hence, the ATG7 gene was selected as a candidate gene to explore its specific function in the development of OS cells, specifically the role of ATG7 in affecting the oxidative stress reaction and ferroptosis process in OS cells.

Notably, the role of ATG7 in regulating tumor progression might be controversial. For example, ATG7's antineoplastic role could suppress tumorigenesis by accelerating tumor cell death in non-small-cell lung cancer and colorectal cancer [59, 60]. ATG7 was linked to better outcomes in renal carcinoma and triple-negative breast cancer [61, 62] while promoting the progression of hepatocellular carcinoma and myeloid leukemia instead [63, 64]. The findings in this study showed that the downregulation of ATG7 significantly enhanced the malignancy of the OS cells, and high ATG7 expression was linked to better survival outcomes, suggesting the protective function of ATG7 in OS patients.

Studies have reported that cellular stress modalities like oxidative stress could induce autophagy [65]. As a key gene of autophagy, ATG7 plays a crucial role in regulating the response to oxidative stress and oxidative stress-induced cell death [66, 67]. Moreover, it was found that ferritin degradation driven by autophagy led to iron accumulation, inducing oxidative stress by the Fenton reaction in cells [15, 68]. Meanwhile, excessive iron accumulation resulted in oxidative damage membrane, triggering the ferroptosis process in cells [14]. The results of the study indicated that silencing ATG7 might inhibit the increase in the oxidizing materials and promote the production of antioxidants, endowing OS cells with a stronger antioxidant capacity when they face oxidative stress. Meanwhile, it also suppressed ferroptosis in OS cells by decreasing the levels of Fe^2+^. These results implicate that ATG7 might promote the ferroptosis of OS cells by modulating oxidative stress. Therefore, ATG7 may be a novel therapeutic target for OS. In addition, autophagy may result in chemotherapy resistance in OS treatment and might serve as a promoter of ferroptosis, while OS patients might benefit from ferroptosis. As the contradictory role of ferroptosis (antitumor) and autophagy (protumor) in OS cells, we believe that using a combination of ferroptosis inducers and autophagy inhibitors might not be advisable when treating OS.

Although one similar study based on 12 FRGs was previously reported [69], differences between the two were as follows: Firstly, the AUC of the previous gene signature was lower than that determined in this study, indicating that the novel FRG signature constructed here has higher accuracy in forecasting the prognosis of the OS patients. Additionally, the number of FRGs was narrowed down to develop a signature (from 12 to 5 FRGs) and improve the predictive ability of the signature, which makes the examination more convenient for clinicians and decreases patient costs. Moreover, all studies constructing predictive FRG signatures for OS patients were only based on bioinformatics methods without any experimental validations, which may make their conclusions less convincing. Finally, the role exerted by the ATG7 gene in oxidative stress and ferroptosis in OS cells was highlighted in this study, which depicted the potential relationship between autophagy and ferroptosis in OS.

The article "Identification of ATG7 as a Regulator of Proferroptosis and Oxidative Stress in Osteosarcoma" was retracted in 2023. Reasons: unreliable results or conclusions; concerns about the data; concerns about the peer review; concerns about the citations.

This study constructed and validated an FRG prognostic signature for OS patients and proposed that ATG7 might promote ferroptosis by regulating oxidative stress in OS. However, it still had some limitations. Firstly, the training and validation cohort sample size was still small, potentially due to the low incidence of OS compared with other tumors. Secondly, this study only focused on ATG7 and explored its specific role in OS, but the effects of the other four genes in OS are still unclear. The function of the remaining 4 genes and their ferroptosis mechanisms in OS cells will be investigated in the future. Therefore, larger sample size and prospective mechanistic studies are needed to validate the results and conclusions of the present study.

## 5. Conclusions

In summary, a novel FRG signature with good accuracy and effectiveness in predicting prognosis for OS patients was constructed. Our results suggested that ATG7 might influence the regulation of oxidative stress, promote ferroptosis in OS cells, and act as a protectively therapeutic target for OS patients. Further studies are warranted to confirm these findings and investigate the fundamental mechanisms of ferroptosis in OS.

## Figures and Tables

**Figure 1:** Tumor classification depending on the 26 ferroptosis-related genes. (a) Univariate Cox regression analysis of 26 FRGs. (b) NMF clustering for 93 osteosarcoma patients based on 26 FRGs. (c) Heatmap depicting the expression of the 26 FRGs in both clusters. (d) The KM curves of both clusters (Log-rank test: ^∗^*p* < 0.05, ^∗∗^*p* < 0.01, and ^∗∗∗^*p* < 0.001).

**Figure 2:** Development of a 5 FRGs-based prognostic signature using the training dataset. (a) LASSO regression analysis of 19 identified FRGs. (b) Cross-validation analysis to tune the parameter selection process in a LASSO regression model. (c) Multivariate Cox regression analysis of 5 FRGs to develop a prognostic signature. (d) ROC curves indicate the prognostic model using 5 FRGs. (e–i) The KM curves of the 5 identified FRGs (Log-rank test: ^∗^*p* < 0.05, ^∗∗^*p* < 0.01, and ^∗∗∗^*p* < 0.001).

The article "Identification of ATG7 as a Regulator of Proferroptosis and Oxidative Stress in Osteosarcoma" was retracted in 2023. Reasons: unreliable results or conclusions; concerns about the data; concerns about the peer review; concerns about the citations.

**Figure 3:** The difference in prognosis and gene expression levels between both the risk groups included in the training dataset. (a) KM curves of patients in the two risk groups. (b) Distribution of individual patients based on the risk scores. (c) Distribution of the survival duration for each patient in the two risk groups (left: low-risk population; right: high-risk population). (d) Heatmap highlighting the FRG expressions in the two risk groups (Log-rank test: ^∗^*p* < 0.05, ^∗∗^*p* < 0.01, and ^∗∗∗^*p* < 0.001).

**Figure 4:** Identifying the risk level as the independent risk factor in a training dataset. (a) Results of univariate Cox regression analysis of OS patients' clinical information, including risk level. (b) Results of multivariate Cox regression analysis of clinical information including risk level. (c) A nomogram that can predict the 1-, 2-, and 3-year survival rates of OS patients. (d) ROC curves examine the predictive ability of the newly established nomogram. (e–g) The agreement between the predicted probabilities and observed outcomes in the nomogram over 1, 2, and 3 years, respectively.

**Figure 5:** Functional analysis of the low- and high-risk groups in the training cohort. (a) GO enrichment analysis based on DEGs between the 2 risk groups. (b) Distinct composition of the immune cells in both risk groups. (c) The scores of 13 immune-related functions to evaluate the immune activities in the two risk groups. (d) Differentially expressed immune checkpoints in the two risk groups (Wilcox: ^∗^*p* < 0.05, ^∗∗^*p* < 0.01, and ^∗∗∗^*p* < 0.001).

**Figure 6:** The difference in prognosis and gene expression levels between both risk groups in the validation dataset. (a) The KM curves demonstrate the distinct overall survival rates in patients from both risk groups. (b) Distribution of patients depending on their risk scores. (c) Distribution of survival duration for every patient (left: low-risk group; right: high-risk group). (d) Heatmap showing the expression levels of 5 FRGs in both risk categories. (e) ROC curves assessed the predictive ability of the 5 FRGs' signature (Log-rank test: ^∗^*p* < 0.05, ^∗∗^*p* < 0.01, and ^∗∗∗^*p* < 0.001).

**Figure 7:** Functional analysis of both the risk groups in the validation dataset. (a) GO enrichment analysis based on the DEGs in both risk groups. (b) Comparing the immune cell components in both the risk groups. (c) The scores of 13 immune-related functions to evaluate the immune activities in two risk groups. (d) Differentially expressed immune checkpoints between the high- and low-risk groups (Wilcox: ^∗^*p* < 0.05, ^∗∗^*p* < 0.01, and ^∗∗∗^*p* < 0.001).

The article "Identification of ATG7 as a Regulator of Proferroptosis and Oxidative Stress in Osteosarcoma" was retracted in 2023. Reasons: unreliable results or conclusions; concerns about the data; concerns about the peer review; concerns about the citations.

**Figure 8:** Analyses of the different groups regarding ATG7 expression. (a) DEGs identified between the low- and high-ATG7 expression groups (blue: downregulated genes; red: upregulated genes). (b) GO enrichment analysis in the differentially expressed ATG7 groups. (c) The different oxidative stress pathways in the two groups.

**Figure 9:** Validation of ATG7 expression and function in OS cells. (a) Relative mRNA expression of 5 candidate FRGs in OS cells and hBMSC. (b) mRNA and protein expressions of ATG7 in hBMSC and MG63 cell lines. (c) The CCK8 assay examines the OS cell proliferation ability after ATG7 silencing and examines ATG7 silencing efficiency. (d) Identifying the influence of ATG7 silencing on OS cell proliferation by colony information assay. (e) Transwell assays examine OS cell migration capability after silencing ATG7 (*n* = 3; *t*-test: ^∗^*p* < 0.05, ^∗∗^*p* < 0.01, and ^∗∗∗^*p* < 0.001).

**Figure 10:** The effect of ATG7 silencing in oxidative stress and ferroptosis in MG63 cells. (a) Cell viability test of ferroptosis-induced MG63 cells after silencing ATG7. (b) Histograms showing the effect of ATG7 silencing in the production of lipid ROS in MG63 cells. (c) Examination of the MDA levels in ferroptosis-induced MG63 cells after ATG7 silencing. (d) Examination of the Fe^2+^ levels in ferroptosis-induced MG63 cells after silencing ATG7. (e) The expression of SOD and FTH1 after silencing ATG7 (*n* = 3; RSL3: 10 *μ*M; time: 12 h; *t*-test: ^∗^*p* < 0.05, ^∗∗^*p* < 0.01, and ^∗∗∗^*p* < 0.001).

## Data Availability

The data used in this study can be found in public databases online. The websites and accession number(s) of the data can be found in the article.

## Supplementary Materials

Supplementary Materials Supplementary Figure S1: the flow chart of this study. Supplementary Figure S2: selecting the best *k* value to classify OS patients into two clusters by NMF method. Supplementary Figure S3: KM curves of another 14 candidate ferroptosis-related genes (*p* ≤ 0.01) that were not included in the prognostic signature. Supplementary Figure S4: identification of risk level as an independent risk factor. Supplementary Table S1: a total of 200 ferroptosis-related genes.
